This article has been retracted.

# Design and Implementation of Mental Health Consultation System for Primary and Secondary School Students Based on Credibility Matching Model

**DOI:** 10.1155/2022/7986850

**Published:** 2022-09-12

**Authors:** Bo Li

**Affiliations:** ^1^Sichuan University of Science and Engineering, Zigong 643000, China; ^2^Philippine Christian University Center for International Education, Manila 1006, Philippines

## Abstract

Primary and secondary schools have the enormous responsibility of developing talent over a hundred years, and they should not only be concerned with the moral, ideological, and cultural development of teenagers but also with their mental well-being. We need to start by making the external environment better, provide in-depth psychological counseling, and support students as they work to continually increase their psychological adaptability in order to promote the healthy development of their personalities. As the epidemic situation in China has now stabilized into a normal state of prevention and control, it is imperative to provide primary and secondary school students with mental health education. In light of this context, this paper develops a browser-server network architecture-based consultation system for the mental health of students in primary and secondary schools. It eliminates the conventional booking mode and substitutes credibility as the characteristic programming parameter. The performance of the original system is improved by the reliability model the most when the parameter is set to 0.2, and the recovery rate rises by 1.32 percent. Compared to the original reliability model, which improved the system's *F* value performance by 0.83 percent, the accuracy rate only declines by 0.68 percent while *F* rises by 0.37 percent. This research is crucial for creating an information campus and raising the standard of psychological counseling.

## 1. Introduction

Future talent should possess a strong physique, a strong personality, and a healthy psychological quality in order to compete effectively in the 21st century. They should also be knowledgeable about modern science and technology and have a wide range of skills. A person's physical and mental development is especially important during adolescence. The interaction between subject and object under the influence of the external environment leads to the psychological development of elementary and secondary school students, with the physiological basis, psychological factors, and environmental influence being the most significant contributors. The same uncertainty is shared by many psychological teachers in primary and secondary schools. There is nothing they can do to take care of each and every student; they are solely in charge of the psychological education of the entire school. The finite energy of teachers and the countless needs of students are in conflict [1]. Primary and secondary school students spent a lot of time at home during the epidemic. On the one hand, they were not accustomed to studying, and there were more issues in the parent-child relationship, which contributed to the decline in physical fitness and in some cases, anorexia, insomnia, and other symptoms. Students who have previously experienced mental health issues will be categorized as having a higher risk of mental problems given the current epidemic situation. In order to prevent their psychological issues from worsening and posing a threat to their safety, schools should offer them prompt and affordable psychological counseling.

Psychological phenomena are essentially the subjective projection of the human brain onto an objective reality, so people's mental health is greatly influenced by the condition of the central nervous system, which has the cerebral cortex at its core. In order to ensure the effective implementation of mental health, the mental health consultation system, which is based on a specific organizational management structure, mobilizes the management resources already in place in schools, such as people, money, things, time, space, information, etc. Not only is management of education the goal, but it is also the means of management [2]. There are many ways that psychology is applied. A psychological test's primary purpose is to assess individual differences in behavior and psychology, as well as behavioral responses and psychological shifts that occur in the same person under various circumstances. As a result, it has many applications and is useful for research. When ANO and others first enroll in school, it is necessary to assess their mental health, create psychological files, incorporate psychological data, and set up corresponding psychological counseling activities [3]. Different from traditional clubs or student organizations, Lilingling has established a variety of mutual aid consultation groups for students, whose goal is to assist students in resolving issues related to their studies, interpersonal relationships, sex, and other areas [4, 5]. To aid primary and secondary school students in developing mental health awareness, maximizing their mental quality, improving their ability to mentally adjust to new situations and adapt to social situations, and preventing and treating psychological issues, Gadomski et al. teach mental health knowledge in a pertinent manner and engage in counseling or consulting activities. Many people will experience different issues during this process. The development of interpersonal relationships is influenced by cognitive, emotional, and personality factors.

The current development trend for mental health education in primary and secondary schools is that many of these institutions have counseling rooms, management institutions for mental health education, or other names [6]. The realization and development of this system not only realized the building of a management system combining various advanced technologies but also realized the efficient demand analysis of exploration results in order to meet the needs of psychological counseling practice in primary and secondary schools. The credibility levels of counselors and counselors to be registered are determined using the credibility requirements of counselors and counselors in the psychological counseling citation system based on credibility matching, using the data with class attribute labels as sample data. In addition, evaluate and judge issues, provide timely guidance to consultants, and aid in issue resolution. The main contributions of this paper are as follows:

1. In view of the shortcomings of the paper-based psychological evaluation method and the abovementioned on-site question-and-answer method, this topic adopts the popular and mature C/S architecture mental health consultation system, based on component technology and middleware, with mental health evaluation as the core, and builds a mental health platform for mental health knowledge dissemination and mental health education.
2. This paper proposes a four-layer access control model based on credibility matching to address the issue of user trust in distributed environments by dynamically calculating user credibility using trusted computing technology. Find the best clustering algorithm, group the consultants and data sets, rank the reliability, and use the reliability to find the best match to maximize resource utilization.

## 2. Related Work

### 2.1. Research on the Mental Health Consultation System

Since the middle of the last century, many foreign colleges and universities have adopted the method of combining computer collaboration with psychological counseling to control their consulting work. Psychological counseling in China is still in the early stage of development, but the overall development speed is extremely fast. At present, both society and schools require better development of psychological counseling services, and many universities globally have made efforts in this respect to establish a more functional psychological counseling system.

Palmer et al. adopted the overall scheme of combining Web page and large database management system based on B/S architecture and ASP.NET technology. The system is mainly composed of several modules, such as background database, user management, psychological intervention management, content management, and psychological testing [7]. Chow et al. mainly use ASP, Access, and other technologies. The database they use is mainly established by Access, and ASP technology, web page calling, and other methods are inserted into the pages to strengthen the scalability of the system [8]. Rothermund et al. designed a network architecture with browser-server mode, which can improve work efficiency and make mental health consultation more regular and efficient [9]. Filho improves the system construction through continuous and in-depth exploration, and strives to develop the system that can provide basic services in the practice of psychological counseling management in primary and secondary schools, and at the same time, it can better enable students to communicate with consultants who conduct counseling services and enhance the service effect of psychological counseling [10].

Mental health service method is a psychological theory and operation technology to correct students' psychological and behavioral problems and promote students' all-round development. The system of mental health service method can better reflect the service level of professionals, schools, and even a country. Song et al. used MD5 (Message-Digest) algorithm encryption and file checking functions to realize the application of system security management and user information security in college students' mental health tracking system, so as to optimize the college students' mental health tracking system and finally improve its security and usability [11]. Zeratsion et al. make use of the existing school websites and campus networks to realize a mental health consultation system for vocational school students based on Internet [12]. This system is a portal system with psychological counseling as its core business and vocational school students as its main clients. With the rapid development of Internet technology, online psychological consultation system has been established. Now there are ready-made examples at home and abroad, and there are quite a few of them. But the problems are also increasing rapidly.

### 2.2. Research Status of Credibility Matching

Ling et al. use *k*-means algorithm to cluster users, and then complete recommendation according to all users or proxy users in the cluster where the target users are located [13]. Hsu et al. solved the problem of data sparsity by principal component analysis. However, this kind of algorithm using matrix dimension reduction not only takes time but also loses some effective scoring information [14]. Paleti et al. put forward a trust calculation algorithm based on project level, topic level, and user outline level, but the calculation of trust is limited by the number of users' scores, so this method needs further improvement [15]. Ghavipour and Meybodi divided attribute acquisition into two steps: the first step is the candidate attribute value acquisition module, and the second step is the candidate attribute verification module. The first step is consistent with the above method. The second step is to use a classifier. For each candidate attribute value, the trained classifier is used to judge which object the attribute belongs to [16].

Wu et al. used the trust estimation method based on Bayesian network and behavior log mining to calculate the prior probability of each attribute trust level according to historical experience, and selected the trust level with the highest conditional probability as the estimation result [17]. Xian et al. proposed a method of judging the matching reliability based on neural network for the normalized edge strength cross-correlation matching algorithm [18]. The back propagation network is used for training, so that the total error of the trained network output is the smallest for the training samples, and the trained network is used to judge the matching reliability. Liu and Chen proposed a Chinese name recognition method based on boundary template and local statistics [19]. This method extracts the boundary template from the tagging corpus, uses the boundary template to roughly delimit the names of people, and then corrects the recognition results according to local statistics and heuristic rules.

## 3. Methodology

### 3.1. Overall Design of the Mental Health Consultation System for Primary and Secondary School Students

Both psychological phenomena and mental health issues are very complex. Relying solely on imported measuring tools frequently falls short of meeting the actual needs of mental health because of social and cultural differences, differences in economic development, differences in educational systems between China and other countries, etc. Health services should create new mental health measurement tools as necessary in addition to introducing foreign measurement tools. Therefore, developmental mental health education should be the main focus of mental health services provided to Chinese students in primary and secondary schools. We will continue to support the development of a localized mental health services system for students in primary and secondary schools in accordance with the principle of gradual progress.

The issue of the shortage of school psychologists and their limited energy is currently being addressed by the psychological early warning system, which is essential. The success of the entire early warning system depends on this, and it serves as its starting point. Through regular communication, this kind of trust relationship is built and gradually reflected. In order to do this, parents and teachers must become experts in working with kids. In light of this, educators and parents should adapt their use of what they have learned, provide prompt assistance in response to students' or children's psychological symptoms, introduce psychological teachers, and make contact with them for expert assistance. This system must be coordinated in order for school psychological education to function as an organic whole.

The functional state of mind is what defines mental health in the most basic sense, and the internal mechanism of mental activities is what determines what that state of mind is. The degree to which various psychological traits have developed and the sophistication of internal mechanisms is, therefore, the primary factor influencing people's mental health. A necessary prerequisite for the healthy development of psychology is the satisfaction of high-level needs, particularly those related to social interaction and self-realization. If satisfaction is insufficient, issues like a lack of motivation, emotional disorder, abnormal reaction, and personality deviation will result. Individual growth may be fueled by this kind of pressure. Stress can also be the root of psychological obstacles or illnesses, although this is more likely when the level of stress is too high or the person's capacity for adaptation is low.

System requirement analysis is the first step in the software development process, which can identify issues early in the system design process and enhance the dialectical rationality of the system. The process of designing and creating requirements documents during the requirement analysis stage can aid in the system architecture and implementation phases later on. However, it is also important to safeguard the system's security as well as the privacy of the students and the security of their personal information. Therefore, it is essential to create a straightforward and effective mental health consultation system.

Every system is fundamentally a data processing system. The information that the system must generate and process determines the information that the system must process, which has a significant impact on the design of the system. As a result, it is necessary to analyze the system's data requirements, which is a crucial component of system analysis. The purpose of this system is to create a service system that can accommodate the current psychological counseling work being done in primary and secondary schools, can assist students in resolving common psychological issues, has a strong expansion effect, and has excellent confidentiality. The system can provide humanized tips, react quickly to user input, and store pertinent data in a database. The system's user interface is sophisticated, uniform in design, and easy to use.

In view of the fact that the system needs to deal with many objects of service function, and has high requirements for the overall security control effect of the system, the C/S architecture is comprehensively selected for construction and treatment. Here, the server chooses an efficient open access control content service system in terms of building functions. The realized communication control is obtained by combining mobile communication processing with Web services, and the overall interactive control ability is good.  Figure 1 shows the detailed architecture layout.

The client created by the system is a member of the resource entrance, where the full scope of psychological counseling work may be done. In order to effectively display information to users, the functional composition is divided into five parts: implementation of the map guidance service, parameter setting service, reservation processing, etc., common function completion, and counseling service implementation. The application layer primarily implements front-end services and back-end micro-services, efficiently harnesses the network's power for information management, and gives schools access to a quick and effective information management mode. The network inquiry system can make student management easier for the school by leveraging the sharing and social aspects of the network.

Through the analysis of users' needs, in order to complete various functions in mental health consultation and analysis, modularization is the function division of application programs. Each module performs a specific function, and these modules are combined into one application program. In the division of modules, try to achieve the independence of modules as much as possible, so that each module can independently complete a specific function, and the interface with other modules is as simple as possible. The psychological system I designed is like the software functional architecture design shown in Figure 2.

The counseling platform publishes news related to psychological counseling through its website and classifies it to make it easier and faster to visit. Consultants can conduct self-test through the test questions provided by the system, and know their most basic psychological state. Counselors can also learn about counselors' psychological state from their answers, so as to be more confident in providing support for future counseling. Through online real-time chat software, excellent long-distance psychological counseling is provided for counselors.

After the function design is completed, you can know how the system functions. Combined with the overall system design, we can roughly analyze the data types that the system needs to store and the functional modules that need to operate some data. The quality of data design has a direct and significant impact on the future coding work of the system, so the design of the database is the key of the whole system design. The beginning of the database design is E-R model, which can be better used to model in the real world and abstract the world from information by analyzing three main elements of the system: entity, attribute, and connection. Draw the E-R diagram related to booking teachers and students according to the teacher center, as shown in Figure 3.

Draw the E-R diagram related to the system information according to the student center, as shown in Figure 4.

Firstly, according to the previous system structure, different local business E-R diagrams are abstracted. Then, use the corresponding rules to merge all local E-R graphs. Finally, we can get the global E-R diagram of the system.

### 3.2. Key Technology Realization of the System

The primary setting for study for students is school, and the educational setting has a significant impact on students' mental health. Since respecting teachers and valuing education is a fine tradition in our nation, and since the relationships between teachers and students are complementary, they must coexist in peace. But in reality, there are some unsettling phenomena in the interactions between teachers and students as a result of the variable quality of some of them. As a member of society, a person will gradually come to accept the influence of his or her surroundings on him or her during his or her development. These environments reflect the long-term accumulation of a particular social history and culture and have clear national and regional characteristics.

The core of the school's psychological early warning system is teachers' psychology, so psychology teachers must be clear about their indispensable role in creating, advancing, and directing the system. Thus, motivation and initiative are essential qualities for psychology instructors. The main goal of mental health education in primary and secondary schools is to promote quality education broadly; enhance the relevance, efficacy, and initiative of school moral education; engage all students; and encourage students to develop healthy psychological qualities. You can schedule a psychological consultation with the teacher's permission, send the teacher a message, change the personal login password, and view the test results with their permission. The foundational information for the archives comes from the student status management system, and the pertinent information about mental health is gathered from online evaluation systems, in-person consultations, counseling, and other sources.

First, we preprocess the data in the reservation system. According to the goal of data mining, we can divide the consultants' and consultants' credibility into *k* categories, and form *k* clusters through cluster analysis. This is the characteristic of K-means algorithm. For example, the ratio of the number of missed appointments to the total number of appointments and the ratio of the number of cancelled appointments to the total number of appointments are relational variables. In clustering analysis, the four attributes are combined to calculate the difference between objects. The formula is as follows:

(1) $$\begin{array}{c} d\left(x_{i},x_{j}\right)=\frac{\sum_{p=1}^{m}\delta_{ij}^{\left(p\right)}d_{ij}^{\left(p\right)}}{\sum_{p=1}^{m}\delta_{ij}^{\left(p\right)}}, \end{array}$$

where *m* is the number of attributes, *i*, *j* are the data objects, and *p* is the attribute variable.

The core of all kinds of matching criteria and algorithms is to obtain the optimal value of one criterion or multiple criteria as the basis of correct matching. After the matching operation, we usually make the following judgment:

The correct matching position is $\left(\hat{x},\hat{y}\right)$, which satisfies the following formula:

(2) $$\begin{array}{c} M\left(\hat{x},\hat{y}|w\right)=\underset{\left(x,y\right)\in \Omega }{\text{OPT}}\left(M\left(x,y|w\right)\right), \end{array}$$

where *M*(·) is a matching criterion, *OPT* is an optimization operator, *w* is a real-time graph, Ω is a search area, and $\left(\hat{x},\hat{y}\right)$ is a matching position in the search area.

It is a method to solve the problem of low recall rate by using the credibility model to supplement the recognition of unrecognized names in the system.

According to the definition of discrimination, let *WN*=*C*_1_, *C*_2_,…, *C*_*n*_ be the name to estimate the character sequence. We think that *WN* is not a person's name only when every word in *WN* is a nonhuman name.

Otherwise, if there is any *C*_*i*_ used as a personal name, the *WN* is likely to be a personal name. Therefore, the name discrimination of the sequence *WN* can be expressed by

(3) $$\begin{array}{c} \text{Diff}\left(WN\right)=1-\left(\prod_{1\leq i\leq n}\left[1-\text{Diff}\left(C_{i}\right)\right]\right). \end{array}$$

In order to prevent a certain pixel (possibly noise) from having too much influence on the overall matching cost when the matching cost is aggregated, the *g*(*C*, *T*) function is used to truncate the *C* values which are too different. The function *g*(*C*, *T*) is

(4) $$\begin{array}{c} g\left(C,T\right)=\left\{\begin{array}{cc} C, & C\leq T,\\ C, & T>T. \end{array}\right. \end{array}$$

Here, *T* is the threshold. Considering that binocular images are collected from different angles, they may be affected by different lighting factors, and if *T* is set too large, it will not play an inhibitory role. If *T* is set too small, the discrimination between pixels is not high.

The credibility matching module mainly involves four categories [20] about how to get the list of consultants. Its attributes include matching thread, matching number, and matching consultant group. The operation mainly includes putting the matching information of consultants into the matching group and deleting it. The class diagram of the credibility matching module is shown in Figure 5.

The mapping relationship between authority and credibility is many-to-many. Here, the mapping relationship between credibility and role is visually expressed by transposing and multiplying authority vector and credibility vector. From this, the calculation formula of the user's credibility can be obtained:

(5) $$\begin{array}{c} \text{UTrust}=w_{2}*\frac{n_{1}}{m_{1}}+w_{3}*\frac{n_{2}}{m_{2}}+w_{4}*\frac{n_{3}}{m_{3}}+w_{5}*\frac{n_{4}}{m_{4}}+w_{1}*t. \end{array}$$

*m*_1_, ⋯, *m*_4_ represent four types of operands: trusted platform, system, security device, and application software, and *n*_1_, ⋯, *n*_4_ represents the number of trusted operations in the four types of operands, where *t* is determined by the system.

Attacks generally consist of a set of false user profiles, which can usually be represented by a vector of *m* dimensions [18]:

(6) $$\begin{array}{c} \text{UP}=\left\{r_{1},r_{2},\cdots ,r_{m}\right\}, \end{array}$$

where *m* represents the number of items in the recommendation system, and *r*_*m*_ represents the user's rating of item *m*.

If the items are randomly selected, the average popularity of the items of the attack profile must be lower than that of real users, so the average popularity can effectively detect such attacks:

(7) $$\begin{array}{c} \text{avg}\left(u\right)=\frac{\sum_{i=I}K_{i}\times P_{u,i}}{\left|I\right|}. \end{array}$$

Here, *u* represents a user; *P*_*u*,*i*_ is 1 when user *u* has scored item *i*, otherwise it is 0; *K*_*i*_ represents the heat of item *i*; *I* represents the set of scoring items of user *u*.

In TF-IDF weighting method, the higher the number of keywords appearing in documents, the higher their weight. The more documents the keywords appear in, the lower their weight. The first formula is as follows:

(8) $$\begin{array}{c} w_{i}=f_{i}*\text{log}\left(\frac{N}{n_{i}}\right), \end{array}$$

where *N* represents the total number of documents, and *n*_*i*_ represents the frequency of keywords appearing in all documents.

Although similar to the single connection method, the longest distance method uses the longest distance between classes when calculating the distance between classes, namely,

(9) $$\begin{array}{c} D\left(m,n\right)=\max\left\{d_{ij}|i\in C_{m,j\in C_{n}}\right\}. \end{array}$$

The clustering algorithm is described, as shown in Figure 6.

In the process of clustering, the vector space model used in this paper is not a numerical vector, but directly takes the value of the attribute as the corresponding value of each dimension of the vector. This grouping method is more suitable for the name disambiguation process based on attribute information. Considering the semantic understanding problem in word comparison, the algorithm uses synonym forest and a group of words to represent words, which alleviates this situation to some extent.

## 4. Experiment and Results

The experiment of this paper mainly investigates the time performance of feature template mining, that is, the influence of various factors on the time performance of frequent node mining. The time-consuming aspect of this algorithm mainly includes three parts: classification, clustering, and feature template mining. Experimental data, this experiment is based on the application of middle school students' elective system. From the middle school teaching database, 4,500 student records, 200 curriculum records, and 15,000 student elective records were selected. Store data in SQL database.

The time-consuming aspect of this algorithm mainly includes three parts: classification, clustering, and feature template mining. Under the condition of constant threshold and constant number of groups, the experiment was carried out with different historical evaluation times, as shown in Figures 7 and 8.

With the same clustering and threshold, the extraction time of feature template increases with the increase of data. The larger the data, the more objects to be evaluated, and the longer it takes. When the number of evaluations is 5000, the algorithm can get the result within 10 minutes, so the algorithm is more efficient and feasible.

This section uses the preliminary results generated by the reference platform to re-identify the names of people, mainly to improve the recovery rate of the whole system. The process is not to re-identify the names of strings that have been identified as individuals. Any processing of names in all texts is just to re-identify the rest of the text. And, the cohesive boundary template is introduced to improve the recovery rate and better ensure the recognition accuracy.  Table 1 shows the recognition results of credibility model with added cohesion and boundary templates.

It can be seen that the increase of the recall rate has a smooth influence on the loss of accuracy rate, and when the value of 0.2 is taken, the credibility model has the greatest improvement on the performance of the original system, with the recall rate increasing by 1.32%, while the accuracy rate only decreases by 0.68%, thus making *F* increase by 0.37%, which is higher than the original credibility model's 0.83% improvement on the performance of *F* value of the system.

We conducted the experiment on the corpus of the real network. There are 4,500 web corpus texts, 3,400 manually labeled attribute texts, and 2,500 attribute texts obtained by the system, with a coverage rate of 74.17%. The experimental results are shown in Table 2.

It can be seen from the table that the performance is gradually improved after weighting the information gain and extending the attributes. This is because in the online corpus, the content of the article is in a free format, and the vocabulary used is relatively free, which will cause inconsistency in language expression. Attribute extension alleviates this inconsistency to some extent. The experimental results show that this method has strong adaptability to corpus. At the same time, this paper improves the existing method and verifies its feasibility.

In order to comprehensively test the influence of the jitter factor on Pearson correlation similarity calculation, it is necessary to simultaneously test its influence on user-based collaborative filtering algorithm and item-based collaborative filtering algorithm. The MAE (Mean absolute error) value of the model in this document is compared with the comparison algorithm, and the experimental comparison is shown in Figure 9. This paper compares the MAPE (Mean Absolute Percentage Error) value between the model and the comparison algorithm, as shown in Figure 10.

According to the experimental results, the proposed model is superior to other models in recommendation accuracy. With the increase of the nearest neighbor number, both MAE index and MAPE index show a downward trend, but the model in this paper is faster and more stable than the original two algorithms. In addition, regardless of the number of nearest neighbors, the algorithm after removing the influence of jitter factor has better recommendation quality than the algorithm before removing the influence.

Using *K*-means clustering analysis, the weighted Euclidean distance from each tuple to each cluster center is found, and finally the new cluster center is determined by redistribution. This process is repeated until the new cluster center does not change any more, as shown in Figure 11.

According to the different weights of each attribute, by comparing the values of the five cluster centers in turn, it can be concluded that the reliability of cluster 2 is the highest, followed by that of the consultant of cluster 1. It is followed by the credibility of consultants in cluster 4, the credibility of cluster 3, and finally the credibility of cluster 5. Then, the corresponding class label is assigned to the consultant's data set.

The living environment and society will undoubtedly have an impact on the mental development stage and mental health of primary and secondary school students since everyone grows and develops within a specific social living environment. The format of mental health education can be based on games and activities in primary schools, activities and experiences in middle schools, and experiences and adaptations in middle schools in order to encourage the close collaboration of educational guidance inside and outside the classroom. By means of the aforementioned tests and analyses, it has been determined that the mental health consultation system developed in this paper can essentially function reliably on a wide range of operating systems with minimal hardware requirements for the installation environment and simple operation and maintenance. We can input, consult, and create statistics quickly and easily in the actual mental health consultation work.

## 5. Conclusions

Implement targeted education in accordance with student psychological development characteristics and the laws of physical and mental development, adhere to educating people, and conduct mental health education in primary and secondary schools. It has been determined through the trial operation analysis of the psychological counseling system for primary and secondary school students that the system increases the productivity of psychological counselors and realizes the website, standardization, and automation of their work. The system essentially realizes a user-friendly interface, practical and convenient operation, and satisfies the fundamental needs of users. Based on credibility and time, booking is more effective when resources are allocated efficiently. It also results in more dependable services. The credibility model performs best when the parameter is set to 0.2; the recovery rate increases by 1.32 percent, the accuracy rate is only decreased by 0.68 percent, and the *F* is increased by 0.37 percent, which is higher than the 0.83 percent of the original credibility model. The psychological well-being of modern primary and secondary school students can be improved to some extent through the psychological health consultation and analysis system, removing the psychological barriers that these students face.

## Figures and Tables

**Figure 1:** System architecture.

**Figure 2:** Software functional architecture design.

**Figure 3:** Teacher's E-R diagram.

**Figure 4:** E-R diagram of students and systems.

**Figure 5:** Confidence matching module class diagram.

**Figure 6:** Clustering process.

**Figure 7:** Influence of the number of clusters on the time of frequent template mining algorithm.

**Figure 8:** Influence of threshold on algorithm time of frequent template mining.

**Figure 9:** MAE comparison.

**Figure 10:** MAPE value comparison.

**Figure 11:** Consultant clustering results.

**Table 1:** Recognition result.

*δ*	Accuracy (%)	Recall (%)	*F* 1 (%)
Benchmark	95.36	83.21	89.13
0.4	95.01	86.74	90.16
0.3	95.23	86.69	90.98
0.2	95.68	86.01	91.35
0.1	94.33	88.64	90.28

**Table 2:** Test results of network corpus.

Test model	Accuracy (%)	Recall (%)	*F* 1 (%)
*K*-means	73.65	60.28	63.17
Bayes	78.91	62.69	68.83
Model of this paper	82.14	68.93	71.48

## Data Availability

The data used to support the findings of this study are included within the article.
